# Automatic Discoid Lateral Meniscus Diagnosis from Radiographs Based on Image Processing Tools and Machine Learning

**DOI:** 10.1155/2021/6662664

**Published:** 2021-04-20

**Authors:** Xibai Li, Yan Sun, Juyang Jiao, Haoyu Wu, Chunxi Yang, Xubo Yang

**Affiliations:** ^1^The Digital ART Lab of School of Software, Shanghai JiaoTong University, Shanghai 200240, China; ^2^Department of Bone and Joint Surgery, Department of Orthopaedics, Shanghai Jiaotong University, School of Medicine, Renji Hospital, Shanghai 200127, China

## Abstract

The aim of the present study is to build a software implementation of a previous study and to diagnose discoid lateral menisci on knee joint radiograph images. A total of 160 images from normal individuals and patients who were diagnosed with discoid lateral menisci were included. Our software implementation includes two parts: preprocessing and measurement. In the first phase, the whole radiograph image was analyzed to obtain basic information about the patient. Machine learning was used to segment the knee joint from the original radiograph image. Image enhancement and denoising tools were used to strengthen the image and remove noise. In the second phase, edge detection was used to quantify important features in the image. A specific algorithm was designed to build a model of the knee joint and measure the parameters. Of the test images, 99.65% were segmented correctly. Furthermore, 97.5% of the tested images were segmented correctly and their parameters were measured successfully. There was no significant difference between manual and automatic measurements in the discoid (*P*=0.28) and control groups (*P*=0.15). The mean and standard deviations of the ratio of lateral joint space distance to the height of the lateral tibial spine were compared with the results of manual measurement. The software performed well on raw radiographs, showing a satisfying success rate and robustness. Thus, it is possible to diagnose discoid lateral menisci on radiographs with the help of radiograph-image-analyzing software (BM3D, etc.) and artificial intelligence-related tools (YOLOv3). The results of this study can help build a joint database that contains data from patients and thus can play a role in the diagnosis of discoid lateral menisci and other knee joint diseases in the future.

## 1. Introduction

Discoid lateral meniscus is an anatomic variant in the knee exhibiting a greater area of the tibial plateau than the normal meniscus. According to studies, having a discoid lateral meniscus increases the possibility of meniscal tears, which leads to symptoms such as pain, clicking, swelling, articular block, limited knee extension, meniscal instability, and the formation of meniscal cysts [1]. Discoid lateral meniscus is relatively common in Asia, and the diagnosis of discoid lateral meniscus needs to take the patient's symptoms and magnetic resonance imaging (MRI) results into consideration. The use of MRI, however, shows several disadvantages during operation. Not every primary hospital may have the capabilities to perform MRI, and even in large general hospitals where MRI is a common tool for diagnosis, patients still suffer from the inconvenience of waiting to make reservations. In addition, MRI has contraindications for patients with magnetic metallic implants or claustrophobia. These factors all contribute to the need to diagnose discoid lateral meniscus on radiographs, which are more popular and convenient and have fewer side effects compared to MRI.

In a previous work [2], a new method to diagnose discoid lateral menisci on radiographs was presented. Several geometric distances and angles were measured from the anteroposterior view of plain knee radiographs, as shown in Figure 1, to identify significant differences between normal and abnormal knees. As a result, significant differences were found in the following parameters: height of the fibular head (HFH), lateral joint space distance (LJSD), height of the lateral tibial spine (HLTS), distance from the lateral tibial spine to the lateral femoral condyle (DLC), chordal distance of the femoral condyle (CDLF), HFH/LJSD, and LJSD/HLTS.

Automating the calculation of LJSD/HLTS using software would be advantageous because this ratio was found to have the largest significant difference between patients who were diagnosed with discoid lateral menisci and normal individuals. Similar studies on radiograph image processing and computer-assisted knee joint analyses were carried out before. Kalinosky et al. [3] developed a detailed method to quantify the tibiofemoral joint space on radiographs using image processing tools to build a spatial model of the knee joint. Other works focused on diagnosing osteoarthritis on knee radiographs, such as the work of Shamir et al. [4], which used several image classification tools to describe features of knee radiograph images, and the work of Lee et al. [5], which used an active shape model to calculate the geometric parameters of the knee joint. Other studies that used an active contour model to locate and segment the region of interest on radiographs were also performed, such as the work of Chen et al. [6], which segmented the patella from knee radiograph images, and Anitha and Prabhu's work [7], which quantified the spinal curvature on radiographs. In recent years, machine-learning-based research has been performed: Zhou et al. used a deep convolutional neural network to obtain a two-dimensional segmentation of a lateral-view knee radiograph [8]; Tiulpin et al. developed a computer-assisted knee osteoarthritis (OA) diagnosis method, which used a deep Siamese convolutional neural network to automatically score the knee OA severity [9]; and Menchon-Lara and Sancho-Gomez's work automatically evaluated carotid intima-media thickness on radiographs [10].

The method to diagnose discoid lateral menisci on radiographs was based on some of the trivial shapes of bones in the knee joint, such as the height of the lateral tibial spine and the shape of the lateral femoral condyle. These features were reflected as graphic details in radiograph images. Therefore, a conservative strategy is preferred, especially when selecting preprocessing tools. When noises are removed from the image, there is also the risk that information of the trivial parts in the image may be lost. Our implementation tried to ensure that no information of edges in the image would be lost. After preprocessing, a well-designed algorithm analyzes the image. By analyzing the overall distribution of the edges and the orientation of each specific edge, high-level features of the knee joint were employed to locate the femur condyle and tibial plateau in the image. Feature points and lines were then drawn in the image, each regarding an important anatomic position of the knee joint. These feature points and lines became the geometric foundation of the parameter calculation. Procedures of the software are demonstrated in Figure 2. The value of the parameter, as indicated in a previous work, differed significantly between normal knee radiographs and abnormal ones [2]. This finding proves that the software automation of the new method is feasible. In addition, the feature points and lines can be stored as personal information of the patient because they contain a geometric description of the femur condyle, tibial plateau, and tibial spine. Databases can thus be built to help record the data of patients, and data could possibly be used to diagnose other knee diseases.

## 2. Materials and Methods

From September 2017 to March 2020, 70 consecutive outpatients (70 knees) who were diagnosed with discoid lateral menisci (discoid group) by MRI were enrolled in the study. Control subjects were selected by a one-to-one matching method with the matching of age and sex (control group). The control patients demonstrated normal medial and lateral menisci on MRI, regardless of other intra-articular pathologies. The discoid group consisted of 43 men and 27 women, with a median age of 33 years (range 20–67 years). The control group consisted of 51 men and 39 women, with a median age of 35 years (range 21–69 years). All patients and controls underwent a standardized knee radiograph that was a nonweight bearing anteroposterior view with a tube (GE Difinium 6000DR, United States) to film a distance of 110 cm. Each plain radiograph was evaluated from the anteroposterior view. All radiographic studies were reviewed by two experienced musculoskeletal radiologists who were unaware of the MRI findings, clinical history, and initial radiographic interpretations. All the measurements were performed on an Advantage Workstation (General Electric Company, United States) using a mouse-point cursor and an automated computer calculation for the distance and angle as described in previous work [2]. The accuracy of distance measurement was 0.01 mm and angle measurement was 0.01°. The figures were rounded to one decimal. The institutional review board of Shanghai Jiaotong University School of Medicine Renji Hospital approved the study protocol (No. KY2019-012) and granted exemption for patient consent.

A total of 160 images from normal individuals and patients who were diagnosed with discoid lateral menisci were included in this study. The software accepts a single image as an input without knowing any specific information about the patient. The software will then try to analyze the image and calculate several parameters, including an important ratio LJSD/HLTS [2].

The software comprises two parts. The first is the preprocessing phase, in which information will be taken from the image. Whether the lateral part of the knee joint is on the left side of the image or on the right side will be decided. The femoral axis and tibial axis will also be determined. Then, YOLOv3 (https://pjreddie.com/darknet/yolo/), an object-detection tool based on machine learning, is used to segment the knee joint from the original image [11, 12]. A median filter, i.e., block-matching and three-dimensional (BM3D) filter, and histogram equalization will be applied to the segmented image for enhancement and removal of noise. The algorithm is implemented with python, using OpenCV 3.4.3 (https://opencv.org/), a state-of-the-art software library for image processing tools [13].

The second part is the measurement phase. In the segmented knee joint image, the femoral condyle will be found by analyzing the distribution of all edges. The femoral condyle becomes the base to find other feature points, including the tibial spines and tibial plateau. When all feature points are found, several lines are drawn on the image, and the calculation is automatically performed. The result of the calculation corresponds to several important parameters mentioned in the previous work, which can signify the discoid lateral menisci of the patient.

### 2.1. Image Segmentation

Raw radiograph images were received as the input of the software, as shown in Figure 3.(a)

We used YOLO to detect and segment the knee joint from the original radiograph images. YOLO is a state-of-the-art, real-time object-detection system based on machine learning [11, 12]. YOLO is feasible for the real-time detection of objects in videos and static images. YOLO frames object detection as a regression problem to spatially separated bounding boxes and associated class probabilities, using a single neural network to predict bounding boxes and class probabilities directly from full images in one evaluation. Traditional object-detection methods, when compared with YOLO, suffer from lower accuracy and failure in images that include multiple objects.

A total of 160 actual X-ray images were selected to fine-tune a pretrained YOLO model. The training process took several hours on an up-to-date machine with GeForce GTX 1080 Ti GPU. Other features of the machine, such as CPU and operating system, will not affect the process of training in any way because only GPU is used for calculation; therefore, their specifications are not listed. The training parameters are listed in Table 1. The same number of real images was tested by the trained network, and we obtained a satisfying result with a success rate of 99.65% in predicting a knee joint; furthermore, none of the predictions were a false positive. As demonstrated in Figure 3(b), the region in the red box is predicted as a knee joint with a probability of 95%. Our fine-tuned model not only performs well in good-quality X-ray images but also on images with flaws and on images including more than one knee.

### 2.2. Image Preprocessing

To enhance the segmented image and remove noise, median filter, histogram equalization, and BM3D filter were applied [14]. In our test, simply using a median blur in the preprocessing phase can reach satisfying results on almost all the images. This process benefits from our measurement algorithm, which is robust against errors in edge detection. However, in some extreme cases, histogram equalization is needed. Histogram equalization was only used when the original image was in extremely low contrast. The total number of edges in the image was counted after the image enhancement phase. If very few edges were detected, the program will abort the current process, use histogram equalization to enhance the image, and then retry. In other normal cases, histogram equalization was not used because it may also enhance noise, and a BM3D filter was used instead.

### 2.3. Measurement

After the preprocessing phase, the measurement of parameters started. First, a Canny edge detector was applied to the image. The canny edge detector is a frequently used algorithm for edge detection [15]. It scans the whole image to calculate the gradient of each pixel and then recognizes high-gradient pixels as possible edges. It then conducts some overall checking and filtering to eliminate false edges, using a pair of parameters provided by the user. In our case, two different groups of parameters were prepared for the Canny detector, (20, 80) and (20, 90), based on the tested image. These parameters indicate the threshold to filter false edges. If one parameter pair fails, similar to what is done in histogram equalization, the software will abort, then switch to another group of parameters, and retry. In all of our cases, this retry strategy of edge detection reached a satisfying result. A satisfactory result of edge detection is shown in Figure 4(e).

To measure the parameters, we started with finding the femoral condyles. All edges in the image were scanned and analyzed to find the POFB edges. An edge that matches the following requirements was recognized as part of the whole femur boundary (POFB): (a) the edge is significantly longer in the horizontal direction, and (b) there is no other edge that lies above it and overlaps with most of the horizontal region it covers. POFB edges can either contain multiple edges or a single edge. If multiple POFB edges are found, all of them will be considered POFB; thus, they will be connected as a new single edge. The new edge is considered to be the upper boundary of the knee joint. In cases in which the quality of the original image was remarkably good, only one POFB edge will be found, and the POFB edge will be naturally considered the upper boundary of the knee joint.

After the upper boundary of the knee joint is found, two local minimum points of the boundary will be marked as the up-left and up-right feature points. The result of finding the femoral condyle boundary and up-left and up-right feature points is demonstrated in Figure 4(f).

Next, two tibial spines were identified. Again, a requirement-matching strategy was used. First, all tip tops in the image were identified. A tip top is defined as a local maximum point of an edge. Consider a single edge (*X*, *Y*) as a pair of coordinates of a point on this edge, and for all the points on this edge, *y* = *F* (*x*). A point (*X*, *Y*) was considered as the tip top if

(1) $$\begin{array}{c} Y=\max\left\{F\left(X-K\right),F\left(X-K+1\right),\ldots ,F\left(X\right),\ldots ,F\left(X+K-1\right),F\left(X+K\right)\right\}, \end{array}$$

where *K* is a constant value determined by the horizontal distance between the up-left feature point and the up-right feature point. Tip tops that are higher than the femur boundary or that are located at the end point of any edge are then removed. A pair of tip tops that matches the following requirements are selected as two tibial spine feature points: (a) they are far away enough from each other, (b) they do not pass the up-left and up-right feature points in the horizontal direction, and (c) they are approximately symmetrical about the axis of the femur. The result of finding the tibial spine is demonstrated in Figure 4(g).

Finally, the baseline of the tibial plateau was identified. From an anteroposterior view, the baseline of the tibial plateau can be defined as a line between the left border of the tibial plateau and the right border of the tibial plateau. Consider a single edge (*X*, *Y*) as a pair of coordinates of a point on this edge, the set of all *x* values on this edge is *S*, and *y* = *F* (*x*). A point (*X*, *Y*) is considered likely to be a border point of the tibial plateau if it is defined as follows:

(2) $$\begin{array}{c} B\left(x\right)=F\left(x\right)*\;\cos\;\theta -x*\;\sin\;\theta ,\\ B\left(X\right)=\max\left\{B\left(X\right),X\in S\right\}, \end{array}$$

where *θ* stands for a specific angle. Imagine putting a ruler on the image and moving the ruler toward the border of the tibial plateau until it finally has a tangent point with the border. This tangent point is recognized as the border point, and *θ* stands for the degree of incline of the ruler. When finding the left edge of the tibial plateau, *θ* can be set as 45°. When finding the right one, it can be set as 135°. Tangent points that go above the femoral condyle baseline are removed, and two tangent points are identified, each corresponding to a value of *θ*. Then, we needed to shift the two tangent points on their original edges to fix deviation. The gradient of the original edge at the tangent point was checked. If the slope is too steep at the border point, it will be shifted inward to find the inflection point where the vertical edge of the tibial boundary connects with the horizontal edge of the tibial plateau and vice versa. After shifting on its original edge, two feature points of the tibial plateau can be determined, and the baseline of the tibial plateau can be drawn. The baseline of the tibial plateau is shown in Figure 4(h).

Now, we have all the necessary information for calculating the parameters. The LJSD is defined as the distance from the upper lateral femoral condyle feature point to the baseline of the tibial plateau. The HLTS is defined as the distance from the lateral tibial spine tip top point to the baseline of the tibial plateau. The ratio of LJSD to HLTS is also calculated automatically as it is a simple division, and this ratio is provided by the software output as the final result of the software-based automatic diagnosis, shown in Figure 4(i).

### 2.4. Statistical Analysis

Differences between groups were evaluated with paired samples *t* test. A *P* value ≤0.05 (two-tailed) was considered statistically significant. All data were analyzed with SPSS (SPSS 24.0, IBM Inc., Somers, NY, USA).

## 3. Results

In Table 1, YOLOv3 training parameters and results are listed. The first four parameters are specific to the neural network. Prediction rate means the ratio of knee images correctly recognized and segmented, and misprediction rate represents the proportion of images for which YOLOv3 successfully provided a result, but the region of the result was incorrect.

Seventy radiographs of patients who were diagnosed with discoid lateral menisci and ninety radiographs from persons without the diagnosis were included in manual or automatic measurement groups. There was no significant difference between manual and automatic measurements in both the discoid group (*P*=0.28) and control group (*P*=0.15). The mean and standard deviations of LJSD/HLTS were compared with the results of manual measurement, as shown in Table 2.

As mentioned previously, the algorithm was divided into two phases, image segmentation and parameter calculation.  Table 3 shows the success rate of each phase. Of the test images, 99.65% were segmented correctly. Furthermore, 97.5% of the tested images were segmented correctly, and the parameters were measured successfully, thus providing necessary information and a software result for the diagnosis.

## 4. Discussion

The most important findings of our previous study are high sensitivity, specificity, and receiver operating characteristic curve area of the LJSD/HLTS and HFH/LJSD between plain radiographic findings from discoid lateral meniscus patients and normal controls [2]. The results of the HFH/LJSD and the LJSD/HLTS showed a positive impact on the diagnosis of the discoid lateral meniscus in this research, which demonstrates that the diagnosis of discoid lateral meniscus using radiographs is feasible and that MRI can be partly replaced by plain radiographs without influencing the final diagnostic results. For patients with the discoid lateral meniscus, diagnosis using radiography is feasible, especially using the HFH/LJSD or the LJSD/HLTS. In this study, we choose LJSD/HLTS for the automatic calculation using a series of software.

Abnormal situations of radiograph images need to be taken into consideration. Some of these situations were solved in our implementation, such as disconnected edges and overall low contrast. Nonetheless, other situations are worthy of attention, such as the situation in which the tibial spine crosses over the femur on the radiograph image, which our algorithm is unable to address. However, the crossing over of the tibial spine and femur can be a sign that the possibility of having discoid lateral menisci is very low, which relieves us from addressing such sophisticated crossover situations. Another situation that should be addressed is the disturbance of the patella.

The BM3D filter performed well in removing noises while keeping details in the image. BM3D is a nonlocal filter for image denoising, which searches for similar blocks in the whole image and builds a 3D data array to distinguish shared details from random noises inside the group [8, 16, 17]. To estimate and rebuild a single block in the group, all similar blocks in the group were used. BM3D has a relatively high computational cost, but it is one of the best tools for image denoising. A median filter is known as one of the basic image processing tools, which simply blurs the whole image to remove pixel values with excessive variation (named salt and pepper noise) when compared locally with other pixels around it. Histogram equalization augmented the whole image by making light areas lighter and dim areas dimmer. BM3D filter recognized shared patterns in the image (e.g., veins on the bone) and augmented these patterns collaboratively to make these image-specific features clearer. Thus, BM3D is very effective in removing stripes and veins on the femur condyle and tibia [16–18]. We have mentioned above that the loss of detail is an unsatisfactory result of image enhancement. However, BM3D performs well in keeping details in the image. It primarily removes large-scale random noises from the image, which are not of concern.

As mentioned in related work, there are several other technical options to achieve a similar goal of automatic diagnosis of certain disease from radiograph images, including feature point, active shape model, and full machine learning, which not only recognizes region of interest but also performs the measurements automatically [11, 12, 18]. We used a two-phase algorithm, which separated machine-learning-based region of interest recognition and parameter measurement because doing so has several advantages compared with the other options. Generally, feature point or other traditional CV (Computer Vision) algorithms are fixed-step structural tools, which are likely to introduce manual operations from software users, which is what we aim to avoid. Also, structural algorithms are not robust against variation of images such as position and rotation of the knee. The active shape model has been proved feasible for radiograph image analysis, but it is too costly to be used and tune. In contrast, a full machine-learning method sounds promising, but it will require an amount of data, which is much larger than what we can currently obtain. Moreover, the internal phases of a neural network are a black box, so the process of measurement and calculation will not be as clear and convincing as that of the two-phase algorithm. Other parameters mentioned in previous work [2] can also be calculated based on our algorithm, although this has not been addressed in this article. To locate the fiber head and measure the inclination of certain edges of the bone and to build a spatial model of the knee joint, more artificial intelligence (AI) tools may be included in future research.

In conclusion, we believe that this is the first study where machine learning was used to diagnose discoid lateral menisci using radiograph images. This new method can be automated, as tests on its software implementation had acceptable results. As a result, it might be possible to diagnose discoid lateral menisci on radiographs with the help of radiograph-image-analyzing software and AI-related tools. Noticeably, machine learning had been used in this study and had satisfactory results. Therefore, this study can become the basis of future research that aims at AI-assisted knee and other joint disease diagnoses. In addition, the results of this study can help build a joint database that contains data from patients and thus can play a role in the diagnosis of discoid lateral menisci and other knee joint diseases in the future.

## Figures and Tables

**Figure 1:** Geometrical definitions of the parameters: height of the fibular head (HFH) from the imaginary tibial joint line to the tip of the fibular head, the lateral joint space distance (LJSD) from the imaginary tibial joint line to the lateral femoral condylar joint line at its midpoint, the height of the lateral tibial spine (HLTS), the height of the medial tibial spine (HMTS), the distance from the imaginary tibial joint line to the tip of the lateral intercondylar spine, and the distance from the lateral tibial spine to the lateral femoral condyle (DLC).

**Figure 2:** Proposed software pipeline.

**Figure 3:** (a) Original radiograph image of the knee joint. (b) Result of the segmentation using YOLO.

**Figure 4:** (a) Original image. (b) Image after applying the BM3D filter. (c) Image after applying a median filter. (d) Image after histogram equalization. (e) Satisfactory result of edge detection. (f) Result of finding the femoral condyle boundary and up-left and up-right feature points. (g) Result of finding the tibial spine. (h) The baseline of the tibial plateau (*θ* > 70°). In this case, shifting is visible on the right border point, as it differs from the right tangent point. (i) Putting everything together. The LJSD and HLTS are drawn on the image. In this case, LJSD/HLTS = 1.325.

**Table 1:** YOLO training parameters and results.

Hyperparameters and results	Value
Batch size	5
Learning rate	0.001
Epoch	100
Momentum	0.9
Prediction rate	99.65%
Misprediction rate	0.00%

**Table 2:** Mean, range, and standard deviations (SD) of LJSD/HLTS.

	Control group (*N* = 90), mean ± SD (95% CI)	Discoid group (*N* = 70), mean ± SD (95% CI)
Manual measurement	0.7 ± 0.2	1.1 ± 0.2
Automating measurement	0.7 ± 0.2	1.0 ± 0.3
*P* value	*P*=0.28	*P*=0.15

**Table 3:** Success rate of each phase.

Phase	Success rate (%)
Image segmentation	99.65
Parameter calculation	97.5

## Data Availability

The data used to support the findings of this study are available from the corresponding author upon request.
